# Diagnostic Imaging Analysis and Care of Patients with Endomyocardial Fibrosis Based on Wireless Network Smart Medical Application

**DOI:** 10.1155/2022/2808889

**Published:** 2022-03-23

**Authors:** Zaomei Chen, Jingya Wen

**Affiliations:** ^1^Emergency Surgery, The 9th Hospital of Wuhan, Wuhan 430081, China; ^2^School of Nursing, Tongji Medical College Huazhong University of Science and Technology, Wuhan 430000, China

## Abstract

The heart is one of the most important organs of the human body, but in recent years heart disease has become one of the human health killers and this paper explores endomyocardial fibrosis, which is a common cardiomyopathy, commonly seen in infants and children, and refers to a diffuse elastic fibrous disease of the endocardium. The purpose of this paper is to explore the diagnostic imaging analysis and care of patients with endocardial heart machine fibrosis using wireless network intelligent medical technology, aiming to provide a new power basis for the treatment of the disease in related patients. This paper proposes a new endocardial segmentation algorithm that aims to process image information using image features, intervene in image noise reduction and smoothing, etc., and use image grayscale values to confirm cardiac cavity grayscale values as a basis for physicians to make certain judgments for the diagnosis of patients with endocardial machine fibrosis. The experimental results show that the atrial fibrillation group is distinctly higher compared to the sinus rhythm group, with values remaining between 25 and 39, which is a significant advantage compared to other methods.

## 1. Introduction

With the continuous improvement of economic level, the living environment around us is also changing, and problems such as serious air pollution are common. Due to the deterioration of the natural environment and the lack of immunity of human body, more and more people are suffering from congenital or acquired heart diseases. The main symptom is the irregularity of the heart's bruit during the cardiac cycle, resulting in problems with the heart's ejection function. Furthermore, studies have demonstrated that myocardial fibers have the double helix structure of the myocardial theory and that there is a clear correlation between the contractile and diastolic forces of myocardial fibers. If the patient is in this state for a long time, more serious heart diseases are likely to develop. Although myocardial fibrosis is a serious killer at present, the traditional diagnostic methods have certain limitations and damage the heart specimen to a certain extent, and the diagnostic results have certain subjective characteristics, so the diagnostic results are inaccurate; in this context a new diagnostic method is urgently needed to provide new treatment pathways for patients with myocardial fibrosis.

The use of wireless network intelligent medical can greatly overcome the shortcomings of traditional diagnostic means, and the design of endomyocardial segmentation algorithm can be automated to overcome the technical limitations of traditional segmentation methods; it can provide therapeutic guidance and help for the treatment of endomyocardial fibrosis by exploring the electrophysiological phenomena of the heart and the structural problems of the heart and making some changes in a targeted manner.

This paper achieves full automation in the analysis and diagnosis of patients with endomyocardial fibrosis using wireless smart net medical compared to traditional endomyocardial cutting techniques, overcoming the traditional method of treating all proportions as a normal heart, and being able to calculate the volume of the heart chambers in the diseased heart during mathematical modeling.

## 2. Related Work

Because endomyocardial fibrotic disease is so damaging to human health, but there is still no scientifically valid means to effectively diagnose it, it has prompted a large number of researchers to explore it in recent years. Münch used three-dimensional whole-mount imaging to reveal the highly dynamic endocardium during cardiac regeneration, including changes in cell morphology, behavior, and gene expression. He explored two important endocardial molecules, Serpine1 and Notch, and found that they are implicated in different aspects of endocardial regeneration, with Notch signaling regulating the expression of developmental genes and characteristics of endocardial maturation; in addition, Notch manipulation interferes with the attenuation of the inflammatory response and the proliferation and dedifferentiation of cardiomyocytes; Serpine1 is strongly expressed early in wound endocardium expression, with reduced expression at later time points, and these probes laid the groundwork for the initial expansion of the endocardium [1]. Zhang has identified many roles for the endocardium in cardiac development, disease, and regeneration with genetic lineage tracing techniques. In addition to the well-known heart valves formed by the transition from endothelial to mesenchymal cells, their fate mapping studies using mouse models showed that multiple cardiac cell lineages also originate from the endocardium, with a variety of different cell types originating from the endocardium during cardiac development, disease, and regeneration, and that the fate of these multiple cells underpins the unprecedented role of endocardial progenitor cells in cardiac function, pathological development, and regeneration role. Studies have shown that developmental mechanisms can be redeployed and reproduced in promoting the development of cardiac disease as well as cardiac repair and regeneration, making it important to understand the mechanistic regulation of the endocardium [2]. Walters used animal models to determine the extent and spatial distribution of endocardial-epicardial dissociation (EED). The experiment used 16 pigs to simultaneously conduct endocardial and epicardial mapping using a 32-electrode grid catheter. Six pigs with rapid atrial pacing-induced atrial remodeling were included, and three right atrial (RA) and three left atrial (LA) regions were mapped during sinus rhythm, atrial pacing, acute or persistent AF, and AF in the presence of pericardial acetylcholine, and offline phase analysis was performed using custom software for unipolar electrogram recordings over 10 seconds, including regional activation patterns on paired surfaces and each matching. The transient phase at each matched electrode location revealed that the average distance between matched endocardial-epicardial electrode pairs was 4.4 ± 1.8 mm, and no rotational activations with ≥3 full rotations were seen during atrial fibrillation episodes [3].

Jiang proposed an energy-efficient multicast routing method for multihop wireless networks for smart medical applications. They investigate the problem of energy-efficient multicast routing in multihop wireless networks for medical applications, point out that energy consumption has become a major issue for the sustainability of communication networks, and argue that performing energy-efficient communication is an important research topic for achieving green communication in wired and wireless networks, and that this problem can be solved by implementing energy-efficient multicast routing methods for networks in multihop wireless networks for smart medical applications. Jiang D proposed three channel assignment strategies to achieve maximum network connectivity through omnidirectional and directional antennas and corresponding algorithms for channel assignment to all cognitive users in cognitive wireless networks. In their experiments they take maximum network connectivity as an optimal goal to build our collaborative channel assignment model and assign the idle channels to the bottleneck nodes considering the channel idle state and transmission radiation status of the cognitive users and then assign the appropriate channels to all other cognitive users as much as possible, which is proved to be effective by experimental simulations [4]. Xu proposed a method using Rabin cryptosystem and chaotic graph scheme for wireless medical sensor networks (WMSNs) in smart medical applications and used several widely accepted security analysis methods to verify the correctness and security of the scheme. Among them, Burrows-Abadi-Needham logical proof confirms the completeness of the scheme and the analysis results show that the scheme is able to resist potential attacks and provide various security properties to be securely applied in wireless medical sensor networks (WMSNs) for smart healthcare [5]. Sohn proposed a new cross-layer QoS provisioning strategy for wireless multimedia sensor networks (WMSNs). The QoS routing problem with multiple objectives is identified as NP-complete, which discovers near-optimal QoS routes by using an evolutionary genetic algorithm. The medium access control (MAC) layer then classifies the packets, automatically adjusts the contention window according to the QoS requirements, and transmits the data using the routing information obtained at the network layer. In this way, wireless sensor networks (WSNs) are guaranteed for applications in automation, medical imaging, traffic monitoring, and surveillance [6].

Nezlobinsky studied the relationship between the velocity of electrically excited waves in one-dimensional isolated myocardial fibers consisting of sequentially coupled cardiomyocytes and that in the same fibers located in the wall of a three-dimensional anatomical model of the left ventricle for estimating the influence of the structure and anisotropy of the left ventricular myocardium on its electrical activation process, and it was shown that in the three-dimensional myocardial tissue the velocity of the wave front fibers is much higher than in the one-dimensional fibers velocities. The acceleration of the signal is due to the rotation of the fiber orientation within the wall and the position of the excitation wave front relative to that fiber orientation. The observed phenomenon is caused by the proximity of excitable tissue with rotational anisotropy to pseudoanisotropic tissue [7]. Although these theories have been introduced to varying degrees in the analysis and diagnosis of endocardial myocardial fibers by wireless smart grid medicine, they can only be applied to one aspect of the diagnosis and lack comprehensiveness.

## 3. Diagnostic Imaging Analysis and Care Methods for Patients with Endomyocardial Fibrosis

### 3.1. Current Status of Intelligent Medical Research

#### 3.1.1. Current Status of Foreign Research

The U.S. program for intelligent medical technology was launched at the beginning of the last century and was the first to start research on intelligent medical technology, and because of its remarkable results in the medical field, Europe and Japan also started to explore intelligent medical technology, and this technology was first applied to large hospitals, where doctors used intelligent medical instruments to detect patients' vital signs to relieve medical pressure [8]. With the continuous development and advancement of science and technology, internet technology has started to be practical in the medical neighborhood and smart medical technology is also progressing, constantly showing a trend towards portability, making it possible to provide personalized services to family members. American companies were the first to develop wearable telemedicine monitoring systems, where patients wear the device on their bodies and the device can detect the body's ECG signal, and patients can observe their ECG signal through the device. The device stores the collected data and location information in a computer, and the data are analyzed and processed by special software, resulting in a data analysis map for reference purposes [9]. One of the smart wearable devices can detect the state of human joint movement, which allows remote monitoring and supervision of patients who have undergone joint-type surgery, so that the process of going to the hospital can be eliminated and patients can complete their rehabilitation at home, saving the medical resources of the hospital and the cost of treatment for the patient. In addition, one of the ring sensors, which patients can wear on their wrists to achieve pulse monitoring of the patient, also has an alarm algorithm set up to keep the bracelet and the patient under monitoring at the same time [10].

#### 3.1.2. Current Status of Domestic Research

Compared with the research process in Western countries, the exploration of intelligent medical technology in China started late and the depth of research cannot be compared with it. The use of intelligent medicine did not appear until the early 1990s, when the PLA General Hospital conducted a joint consultation with a foreign hospital via remote video [11]. However, until now, the technology has not been used on a large scale in China. A university has developed a small nurse system consisting of a home monitor and a hospital server, which successfully enables patients to monitor their ECG and blood pressure at home and can analyze the data in real time; if the system considers the data abnormal, it will send the abnormal data to the hospital's server, and then an expert will view the abnormal data and organize a consultation. In addition, the Academy of Military Medical Sciences has developed a wearable medical monitoring system, which distributes information-gathering instruments on outerwear, so that if you want to conduct tests, you can directly put on the outerwear. The information collected by this device can be transmitted to electronic devices through a wireless network for easy viewing by medical personnel [12]. The system can achieve both remote monitoring and mobile monitoring. With the development of internet technology, intelligent medical systems have gradually aroused national attention, and currently, intelligent medical-related systems have been used in the market. Using internet technology to monitor the daily life of the guardian and to detect various vital signs of the human body, the system has the ability to notify the nearest hospital and family members if the patient goes out of the guardianship range or has an accident to provide timely assistance to the warded person, which greatly improves the cure rate [13].  Figure 1 shows the intelligent system diagram.

#### 3.1.3. Development Trend

With the development of internet technology, the internet of things technology is applied to various fields such as drug production and anticounterfeiting; according to the drug label, the production source, production date, logistics information, etc. can be read out, which can successfully detect the various links between drug production and drug use. In the area of patient medical records, successfully used intelligent medical systems can also get information about the patient's condition and personal information in real time, so that information can be shared between hospitals in real time [14, 15].

### 3.2. Image Processing

Image processing regarding endocardial myocardial fibers has an important impact on the whole diagnostic process. The acquired images have ripple-like features in addition to noise problems, and if this image can be processed accurately, it will help a lot in the subsequent endomyocardial fibers diagnosis [16].  Figure 2 shows the system diagram of fiber tracking results.

Entropy, originally used to represent the distribution of energy in thermodynamics, has also gained ground within the medical field in recent years, and we define its functional expression as

(1) $$\begin{array}{c} F\left(a\right)=-q\sum_{i=1}^{m}k_{i},\;\ln\left(k_{i}\right), \end{array}$$

in which ∑_*i*=1_^*m*^*k*_*i*_=1， *k*1=*k*2=*k*3=⋯*km*, when F takes the maximum value.

In the image processing process, entropy is mainly used to distinguish the foreground color from the background color, and the main basis for distinguishing the foreground color from the background color is the grayscale value, and there is a big difference between the two in the distribution of grayscale values. We express the expression of the grayscale value as follows:

(2) $$\begin{array}{c} D_{1}\left(a\right)=-q\sum_{i=0}^{q-1}k_{i}\ln\left(k_{i}\right),\\ k\left(i\right)=\frac{g\left(i\right)}{\sum_{j=0}^{q-1}g\left(i\right)}, \end{array}$$

in which *g*(*i*) is the gray value function, *q* is a constant, and *k*(*i*) represents the range of gray values in 0–1.

The entropy of the part larger than the threshold *q* is expressed as

(3) $$\begin{array}{c} D_{2}\left(a\right)=-q\sum_{i=q}^{255}k_{i}\ln\left(k_{i}\right),\\ k\left(i\right)=\frac{g\left(i\right)}{\sum_{j=q}^{255}g\left(j\right)}, \end{array}$$

in which *g*(*i*) denotes the gray value function, *q* is a constant, and *k*(*i*) represents the range of gray values in q-255.

The sum of the two entropies is given by

(4) $$\begin{array}{c} D\left(a\right)=D_{1}\left(a\right)+D_{2}\left(a\right), \end{array}$$

in which *D*(*a*) is maximum and the threshold is the maximum entropy threshold, that is, the threshold that distinguishes the foreground color from the background color.

In the actual processing, the gray value fluctuates very significantly in a small range, and in order to find the peak accurately, the gray map of the image needs to be intervened. We use exponential smoothing method for smoothing, whose function expression is as follows:

(5) $$\begin{array}{c} Y\left(a\right)=\left(1-\beta \right)*Y\left(q-1\right)+\beta *H\left(a\right), \end{array}$$

where *a* represents the gray value, q-1 represents the smoothed value, *H*(*a*) is the original value, and *ß* represents the constant.

Smoothing of images is a very common technique that uses pixel points to calculate the weighted average to calculate the gray value, and the weighted average is its core element, defined as

(6) $$\begin{array}{c} y\left(a\right)=\frac{u}{\partial \sqrt{2\pi }}e^{-\frac{{\left(a-\varepsilon \right)}^{2}}{2\partial^{2}}}, \end{array}$$

in which the Gaussian distribution expectation is *ε*, the standard deviation is ∂, and the standard Gaussian distribution is *ε* = 0 and ∂  = 1.

In practical processing, we commonly use the Gaussian fuzzy two-dimensional Gaussian distribution density distribution function, whose expression is expressed as

(7) $$\begin{array}{c} H\left(a,b\right)=\frac{1}{2\pi \lambda^{2}}e^{-\frac{a^{2}+b^{2}}{2\lambda^{2}}}, \end{array}$$

in which *λ* represents the standard deviation.

The Gaussian blur forms a circular lamp height line on the surface in two dimensions, and defining its radius as *r*^2^=*a*^2^+*b*^2^, the following expression can be derived:

(8) $$\begin{array}{c} H\left(a,b\right)=\frac{1}{2\pi \lambda^{2}}e^{-\frac{a^{2}+b^{2}}{2\lambda^{2}}}. \end{array}$$

In image processing, the method can form a rectangular template; when the center point is larger, the other values are in a large negative growth relationship with the distance to that point. The formula for Gaussian template image processing is

(9) $$\begin{array}{c} S\left(a,b\right)=\sum_{i=0}^{i=n}\sum_{j=0}^{j=n}H\left(i,j\right)*s\left(a_{0},b_{0}\right),\\ a_{0}=a+\left(i-\left[\frac{n}{2}\right]\right),\\ b_{0}=b+\left(j-\left[\frac{m}{2}\right]\right), \end{array}$$

in which *H*(*i*, *j*) represents the point in the coordinates and a is the largest integer.

Using the preprocessed ultrasound image, its characteristics on the gray value map are analyzed and the site to be segmented is confirmed using a threshold value, making the segmentation more precise and the diagnosis more accurate.  Figure 3 shows the flow chart of the endocardial segmentation algorithm.

Curve evolution is described academically as the process by which a smooth closed curve existing in two-dimensional Euclidean space, moving at a certain speed according to its direction, can form a series of curve clusters, and we call this process curve evolution, which we define as

(10) $$\begin{array}{c} \frac{\beta A\left(z\left(c\right),b\left(c\right)\right)}{\beta c}=S\left(z\left(c\right),b\left(c\right)\right)M, \end{array}$$

in which A represents the curve function, *z*(*c*), *b*(*c*) represents the point on the curve with *c* as the independent variable, S represents the curve velocity, *M* represents the curve unit vector, and the curve evolution direction is shown in Figure 4.

When exploring the evolution of curves, it is often necessary to perform formal transformations, and we denote the curve curvature deformation as

(11) $$\begin{array}{c} \frac{\theta A}{\theta z}=\partial k\;M, \end{array}$$

in which ∂ represents a positive constant, *k* represents the curve curvature, and *M* represents the unit normal vector, and in the expression, the constant deformation can be expressed as

(12) $$\begin{array}{c} \frac{\theta A}{\theta z}=\beta M, \end{array}$$

in which *ß* represents the constant and *M* represents the unit normal vector, but the curvature of the previous curve is not taken into account when *ß* is a constant, so anomalies will appear when performing the calculation. This problem was not solved until someone proposed that the level set method could be used on curve evolution, and Figure 5 shows the schematic diagram of level set curve evolution.

We express the distance to the zero-level set curve at the starting arbitrary point by the following functional expression:

(13) $$\begin{array}{c} \beta \left(a,b,t=0\right)=\pm \lambda \left(a,b\right). \end{array}$$

This distance is positive or negative; if the point is inside the curve it is negative and if the point is outside the curve it is a positive distance, so this distance is determined by the position of the point and the specific expression is as follows:

(14) $$\begin{array}{c} \beta \left(a,b,t=0\right)<0,\\ \beta \left(a,b,t=0\right)=0,\\ \beta \left(a,b,t=0\right)>0. \end{array}$$

At any moment, the zero-level set of the corresponding surface of the curve is

(15) $$\begin{array}{c} \beta \left(Q\left(x,y\right),t\right)=0. \end{array}$$

Differentiate it to get

(16) $$\begin{array}{c} \frac{\theta \beta }{\theta t}+\frac{\theta \beta }{\theta Q}*\frac{\theta Q}{\theta t}=0. \end{array}$$

It is known that the zero-level set conforms to the evolutionary curve during the evolution of the curve; by its definition we can obtain

(17) $$\begin{array}{c} \frac{\theta \beta }{\theta a}=\frac{\theta \chi }{\theta x}*\frac{\theta x}{\theta a}+\frac{\theta \beta }{\theta y}*\frac{\theta y}{\theta a}=\frac{\theta \beta }{\theta Q}*\frac{\theta Q}{\theta a}=0. \end{array}$$

When the point is inside the curve, we can express it as

(18) $$\begin{array}{c} M=-\frac{\nabla \theta }{\left|\nabla \theta \right|}. \end{array}$$

Organizing the expressions yields

(19) $$\begin{array}{c} \frac{\phi \theta }{\phi t}=-\nabla \theta *ZM=\nabla \theta *Z*\frac{\nabla \theta }{\left|\nabla \theta \right|}=Z\left|\nabla \theta \right|. \end{array}$$

In summary, the velocity field of the horizontal set satisfies

(20) $$\begin{array}{c} \frac{\phi \theta }{\phi t}=Z\left|\nabla \theta \right|. \end{array}$$

### 3.3. Patient Care

Patient care service refers to the physical or psychological needs in a certain medical environment. As society continues to improve, people's health consciousness is rising and their requirements for care are becoming higher and higher, and patient needs are evolving towards a diversified and dynamic trend. For hospitals, then, accurate awareness of patients' needs is important for improving service quality. In large hospitals, for example, there must be many patients with serious illnesses, which results in many patients and a large flow of people, which brings the problem of a wide range of patient needs. How to meet the reasonable needs of patients and make them physically and mentally happy is an important issue that needs to be solved in nursing, which also directly affects the quality of hospital services [17, 18].

At present, the nurse-patient relationship is facing new threats, and patients' expectations of nurses are getting higher and higher, leading to a greater psychological gap, so patients complain that nurses are not doing their nursing duties, and contradictory to this, there are more and more patients in hospitals, and nurses' work tasks are getting heavier and heavier, and their professional skills and service attitudes are improving [19]. In-depth exploration could find that the emergence of this contradictory situation is mainly because the patient's psychological expectations are too high, and the services they can receive are different from what they expect, resulting in a huge gap, and also because of the task. As a result, nurses cannot accurately identify the needs of patients or cannot meet the needs of patients in a timely manner. Therefore, timely and accurate identification of patients' needs and meeting their needs is the focus of nursing work [20].

## 4. Diagnostic Imaging Analysis and Nursing Care of Patients with Endomyocardial Fibrosis

### 4.1. Experimental Materials

#### 4.1.1. Experimental subjects

Fifty healthy rats with body weight kept near 225 g were taken, and the room was kept at a constant temperature with relative humidity kept above and below 50%, and a number of replacement mice were accurate [21].

#### 4.1.2. Experimental tools

Table 1 shows the instruments and specifications to be used for the experiments, including but not limited to cloxacin tablets, gentamicin needles, paraformaldehyde, and quantitative enzyme assay kits, among others.

### 4.2. Experimental Methods

The mice were randomly divided into surgical group and sham group. Before surgery, the mice were completely fasted, anesthetized before surgery, fixed on the operating table, and connected to ECG and ventilator to prevent abnormal conditions during surgery, and the body temperature of the experimental mice was kept constant. If the electrocardiogram showed abnormal condition, it indicated myocardial infarction, so the heart should be reset immediately, the wound should be sutured, the vital signs should be observed, the ventilator should be withdrawn after the respiration remained stable, and the endocardial model was prepared successfully. The sham-operated group had the same procedure as the operated group, but the ligation step was not required during the delivery line [22, 23].

### 4.3. Experimental Data

Table 2 shows the table of cardiac function status in mice, and according to the data in the table, LVEDD and LVESD were significantly abnormal and IVS, LVEF, and LVFS were reduced in the model and drug groups compared to the sham-operated group [24].

Table 3 shows the status of the effect of the optimized formula with ginseng on serum BNP in endocardial mice. Compared with the sham operation, the model and drug groups were significantly different, and the values of the small and large dose groups were compared with the model group when there was a decreasing trend, and the reference group was coxsartan when there was no significant change in their change values.  Table 4 is the changes of body mass index in mice during endocardial exercise.

As shown in Table 4, no significant changes in the heart rate and weight of the experimental subjects occurred throughout the procedure, but the LVWI in the model group appeared elevated when it was with the sham-operated group as the reference group; there were no significant changes in the drug group when cloxacin was used as the reference group [25].  Table 5 is the effect of hydroxyproline content in endocardial white rats.

As shown in Table 5, when the sham-operated group was used as a reference, the hydroxyproline content of the simulated and drug groups showed a significant increase, and when the model group was used as a reference, the hydroxyproline content of the small-dose group showed no abnormalities, but at this time the high-dose group and the cloxacin group showed a reduced condition [26].

## 5. Diagnostic Imaging Analysis and Care Analysis of Patients with Endomyocardial Fibrosis

### 5.1. Analysis of LVED and LVESD Data

Figure 6 is the status of cardiac function in experimental subjects. It is clearly evident from Figure 6 that the values of LVEDD and LVESD in the high-dose and cloxacin groups showed a decreasing trend if the model group is included as the reference group, and at this moment, the LVS in the drug group, the high-dose group, and the cloxacin group showed an increasing trend in values, and none of the remaining groups showed a significant trend when cloxacin was included as the reference object. LVEDD represents the left ventricular diastolic status, LVESD represents left ventricular systolic status, LVEF represents ejection fraction, and LVFS represents cardiac event short sleeve systolic rate [27].

Figure 7 is effect of adding ginseng to optimize the formula on cardiac function. It is clearly evident from Figure 7 that it can be seen that when the sham-operated group was taken as the reference group, the values of the model group and various drug groups showed an elevated phenomenon; when the model group was included as the reference object; the values of the small-dose group, the high-dose group, and the cloxacin group showed a pairwise decreasing trend; when the cloxacin group was taken as the reference object, the values of the remaining data groups did not show significant changes [28].

### 5.2. Comparative Analysis of SR and AF Cardiomyocytes

Figure 8 is comparison of LAD between patients in SR and AF groups. It is clearly evident from Figure 8 that the left atrial volume appeared significantly enlarged in the group of patients with wind AF, and there were no significant differences between the two control groups in other conditions such as gender, age, LVEFHE, and cardiac function classification. Patients saw a small amount of collagen fibers in the subendocardium and interstitium and no collagen fiber encapsulation in the myocardial bundle, while patients with AF showed more collagen deposition in the subendocardium and interstitium with a small amount of collagen fibers visible [29].

### 5.3. Genetic Analysis of Type I and Type III Collagen

Figure 9 is comparison of the relative expression of type I and type III collagen. It is clearly evident from Figure 9 that the amplification product band of DNALadder with 320 bp was the target gene type I collagen and the amplification product band with 659 bp was the target gene type III collagen [30–32]. The mRNA expression of type I collagen in the atrial tissue was significantly higher in the atrial fibrillation group than in the sinus rhythm group, and the mRNA values of type III collagen showed a higher trend in the atrial fibrillation group than in the sinus rhythm group [33–36].

## 6. Conclusions

Based on previous experience and existing theoretical basis, a new endocardial cutting technique was proposed in this paper. Compared with previous techniques, we performed prior processing of the image to be diagnosed before cutting, transformed the image information into ultrasound image grayscale values, then analyzed according to the grayscale value data features to find the distinguishing points between foreground and background in the image until finding the wave peak position, and finally performed noise reduction process to improve the accuracy of diagnosis. In this paper, the following tasks were accomplished: (1) visualization of the intensity values of myocardial fibers was carried out using the plotting maneuver and the fiber tracking method and marking the direction in the processing. (2) An innovative treatment of endomyocardial cutting technique was performed, which allows automation in designing endomyocardial segmentation algorithms and overcomes the technical limitations of traditional segmentation methods. (3) By exploring the electrophysiological phenomena of the heart and the structural problems of the heart, some changes are targeted to provide therapeutic guidance and help for the treatment of endocardial myocardial fibers. However, due to the limitation of our own ability, there are still many problems to be explored: (1) the results of endomyocardium alone cannot accurately diagnose the patient and determine the cause, necrotic area, and degree of disease, which largely restricts the cure rate of patients. (2) It is hoped that the central path algorithm can be applied to ultrasound images to find the standard cut of the cardiogram through multiple path planning to improve the correct diagnosis rate [37].

## Figures and Tables

**Figure 1:** Intelligent system diagram.

**Figure 2:** Fiber tracking result system.

**Figure 3:** Flow chart of endocardial segmentation algorithm.

**Figure 4:** Curve evolution directions.

**Figure 5:** Schematic diagram of the evolution of the horizontal set curve.

**Figure 6:** Status of cardiac function in experimental subjects.

**Figure 7:** Effect of adding ginseng to optimize the formula on cardiac function.

**Figure 8:** Comparison of LAD between patients in SR and AF groups.

**Figure 9:** Comparison of the relative expression of type I and type III collagen.

**Table 1:** Experimental tools and specifications.

Name	Specification
Gentamicin injection	General
Paraformaldehyde	General
Clozaril tablet	0.1 g/tablet
Ang quantification enzyme	General
BNP quantification enzyme	General

**Table 2:** Cardiac function status of mice.

Group	Fake surgery group	Model group	Low-dose group	High-dose group	Cloxacin group
n	7	7	7	7	7
LVEDD (cm)	0.62	0.83	0.75	0.73	0.81
LVESD (cm)	0.32	0.80	0.63	0.65	0.57
IVS (cm)	0.25	0.17	0.21	0.20	0.23
LVEF (%)	81.17	38.9	45.3	49.8	52.7
LVFS (%)	82.6	39.7	46.3	55.2	53.4

**Table 3:** Effect of endocardial serum BNP.

Group	n	BNP (pg/ml)
Fake surgery group	7	16.7
Model group	7	92.8
Low-dose group	7	77.9
High-dose group	7	63.8
Cloxacin group	7	52.9

**Table 4:** Changes in weight index of endocardial mice doing things.

Group	Fake surgery group	Model group	Low-dose group	High-dose group	Cloxacin group
n	7	7	7	7	7
BW (g)	399	420	403	405	381
HR (beat/min)	400	415	440	450	400
LVWI (‰)	1.21	2.17	1.87	1.74	1.84

**Table 5:** Effect of hydroxyproline content in endocardial white rats.

Group	*n*	Hydroxyproline (*μ*g/mg)
Fake surgery group	4	2.99
Low-dose group	4	13.57
High-dose group	4	11.35
Cloxacin group	4	10.25
Model group	4	14.35

## Data Availability

The data used to support the findings of this study are available from the author upon request.
